The article "The smoking paradox in ischemic stroke patients treated with intra-arterial thrombolysis in combination with mechanical thrombectomy–VISTA-Endovascular" was retracted in 2022. Reasons: errors in the data; errors in the analysis; concerns about the results or conclusions.

# The smoking paradox in ischemic stroke patients treated with intra-arterial thrombolysis in combination with mechanical thrombectomy–VISTA-Endovascular

**DOI:** 10.1371/journal.pone.0251888

**Published:** 2021-05-20

**Authors:** Anna Kufner, Huma Fatima Ali, Martin Ebinger, Jochen B. Fiebach, David S. Liebeskind, Matthias Endres, Bob Siegerink, on behalf of the VISTA-Endovascular Collaborators

**Affiliations:** 1 Center for Stroke Research Berlin, Charité–Universitätsmedizin Berlin, Corporate Member of Freie Universität Berlin, Humboldt-Universität zu Berlin, and Berlin Institute of Health, Berlin, Germany; 2 Berlin Institute of Health (BIH), Berlin, Germany; 3 Klinik und Hochschulambulanz für Neurologie mit Experimenteller Neurologie, Charité-Universitätsmedizin Berlin, Berlin, Germany; 4 Berlin School of Mind and Brain, Humboldt-Universität zu Berlin, Berlin, Germany; 5 Department of Neurology, Medical Park Berlin Humboldtmühle, Berlin, Germany; 6 UCLA Stroke Center, Los Angeles, CA, United States of America; 7 German Centre for Cardiovascular Research (DZHK), Partner Site Berlin, Germany; 8 German Center for Neurodegerenative Diseases (DZNE), Partner Site Berlin, Germany; 9 ExcellenceCluster NeuroCure, Charité-Universitätsmedizin Berlin, Berlin, Germany; Hospital Dr. Rafael A. Calderón Guardia, CCSS, COSTA RICA

## Abstract

**Background:**

The smoking-paradox of a better outcome in ischemic stroke patients who smoke may be due to increased efficacy of thrombolysis. We investigated the effect of smoking on outcome following endovascular therapy (EVT) with mechanical thrombectomy alone versus in combination with intra-arterial (IA-) thrombolysis.

**Methods:**

The primary endpoint was defined by three-month modified Rankin Scale (mRS). We performed a generalized linear model and reported relative risks (RR) for smoking (adjustment for age, sex, hypertension, atrial fibrillation, stroke severity, time to EVT) in patient data stemming from the Virtual International Stroke Trials Archive—Endovascular database.

**Results:**

Among 1,497 patients, 740(49.4%) were randomized to EVT; among EVT patients, 524(35.0%) received mechanical thrombectomy alone and 216(14.4%) received it in combination with IA-thrombolysis. Smokers (N = 396) had lower mRS scores (mean 2.9 vs. 3.2; p = 0.02) and mortality rates (10% vs. 17.3%; p<0.001) in univariate analysis. In all patients and in patients treated with mechanical thrombectomy alone, smoking had no effect on outcome in regression analyses. In patients who received IA-thrombolysis (N = 216;14%), smoking had an adjusted RR of 1.65 for an mRS≤1 (95%CI 0.77–3.55). Treatment with IA-thrombolysis itself led to reduced RR for favorable outcome (adjusted RR 0.30); interaction analysis of IA-thrombolysis and smoking revealed that non-smokers with IA-thrombolysis had mRS≤2 in 47 cases (30%, adjusted RR 0.53 [0.41–0.69]) while smokers with IA-thrombolysis had mRS≤2 in 23 cases (38%, adjusted RR 0.61 [0.42–0.87]).

**Conclusions:**

Smokers had no clear clinical benefit from EVT that incorporates IA-thrombolysis.

## Introduction

It is well-known that smoking has detrimental effects on the cardiovascular system and leads to increased atherosclerosis, ischemic stroke, and myocardial infarction [1]. The so-called “smoking paradox” refers to a better outcome following intravenous thrombolysis (IVT) as well as endovascular therapy (EVT) in smokers following AIS [2–5]. While some attribute this effect to a form of selection bias known as collider stratification bias or index-event-bias which causes an accumulation of otherwise lower risk profiles amongst the smokers [6, 7], others have suggested a more causal effect of smoking, in which smoking leads to increased treatment efficacy of thrombolysis in the setting of acute stroke [2, 3, 5].

The pathophysiology behind the suspected increased treatment efficacy in smokers might be explained by a reduction of endogenous tPA release from endothelial cells in smokers [8, 9]. While this may cause hypercoagulability and increased risk of intravascular thrombus formation [10], these thrombi are likely more fibrin-rich and may thus be more susceptible to exogenous tPA [10–12]. In other words, smoking may modify clot dynamics in such a manner that the efficacy of thrombolysis is increased.

The aim of this study was to perform an interaction analysis of smoking and selected EVTs in a large, homogenous cohort of patients with proven large vessel occlusion (LVO), enrolled in endovascular randomized controlled trials (RCTs). We hypothesized the so-called smoking-paradox of a better functional recovery in patients eligible for EVT with LVO, who receive intra-arterial thrombolysis (IA-thrombolysis) and not in those who undergo mechanical thrombectomy alone.

## Methods

### Ethical approval and informed consent

Ethical approval was obtained for each randomized controlled trial included in this dataset; all patients provided informed consent. Which clinical trial the patients were enrolled in remains anonymous within the VISTA-Endovascular dataset to prevent re-analysis of already completed randomized controlled trials. For specifics regarding ethics approval and informed consent, please contact the VISTA-Endovascular research group.

### Patient population

All data come from the Virtual International Stroke Trials Archive—Endovascular database (VISTA-Endovascular, URL: www.virtualtrialsarchives.org): anonymized data of approximately 1,788 patients with acute ischemic stroke enrolled in endovascular RCTs. Anonymized data were compiled from the archive based on the availability of pre-specified variables of interest for the current analysis. Prior to the data analysis, a project proposal with the pre-defined outcome parameters was approved by the VISTA Steering Committee.

### Clinical and imaging definitions

For this analysis, smoking was defined as active tobacco smoking at the time of stroke, a binary variable to distinguish between current smokers and non-smokers; non-smokers included ex-smokers as well. The site of arterial occlusion was categorized into four groups; internal carotid artery (ICA) only; ICA with involvement of M1 segment of the middle cerebral artery (MCA) or M1 segment only or M1 along with several M2 segments afflicted; single M2 segment only; and other proximal vessel occlusions i.e., proximal occlusion of the anterior cerebral artery (ACA) or M3 segment.

The main outcome of interest was the modified Rankin Scale (mRS; an ordered nominal score ranging rom 0 to 6 with 0 indicating no symptoms and 6 indicating death) assessed 90 days post-stroke on an ordinal scale and good outcome defined as a binary variable (mRS ≤/> 2). Second outcomes of interest included excellent outcome (mRS ≤ 1) and mortality (mRS = 6) also assessed at 90 days. Tertiary outcomes of interest included assessment of daily activities assessed by Barthel Index (BI; an ordered nominal scale that measures performance in activities of daily living) at 90 days, recanalization and reperfusion rates post-treatment, lesion progression, and presence of collaterals assessed at baseline.

Successful recanalization was defined as the Thrombolysis in Cerebral Infarction (TICI) grade 2B or 3 on angiography 24 hour post-treatment [13]. Successful reperfusion was defined as modified Thrombolysis in Cerebral Infarction (mTICI) grade 2B or 3 on 24-hour follow-up scan [14]. The data for collateral status was dichotomized into good (filling of ≥ 50%) and poor (filling of < 50%) of MCA pial arterial circulation on digital subtraction angiography. Lesion volumes were provided by the selected RCTs; lesion progression was calculated in milliliters and specified by the variables relative infarct growth (follow-up lesion volume/baseline lesion volume) and absolute infarct growth (follow-up lesion volume—baseline lesion volume).

### Statistical analyses

For all two-group univariate analyses, Pearson chi-square or Fisher exact test and Wilcoxon-Mann-Whitney U test or Student’s t-test were applied where appropriate. We performed regression analyses for all pre-defined outcome measures and reported unadjusted and adjusted relative risks (RR) or odds ratios (OR) as appropriate for smoking status. Regression analyses were performed in three pre-defined patient cohorts, namely 1) all patients regardless of treatment allocation, 2) patients who received mechanical thrombectomy alone, and 3) patients who received mechanical thrombectomy with IA-thrombolysis. All regression analyses for binary endpoints were performed by generalized linear model (glm) using a modified log-Poisson regression model with a robust error variance to reduce risk of overestimation [15].

Subsequently, we analyzed the individual as well as the combined effects from both smoking and IA-thrombolysis treatment for all binary outcome endpoints. We did so by estimating the RRs for the four patient groups depending on the combined exposure (i.e. non-smokers/—IA-thrombolysis, smokers/—IA-thrombolysis, non-smokers/ + IA-thrombolysis, smokers/ + IA-thrombolysis), always with the non-smokers/—IA-thrombolysis as a reference. This type of analysis assesses whether there is evidence for additive interaction.

For all regression analyses, models were adjusted for age, sex, hypertension, atrial fibrillation, baseline National Institute of Health Stroke Scale (NIHSS), and time to endovascular treatment from symptom onset. All statistical analyses were performed with STATA/SE 12.1 statistical package (StataCorp).

## Results

### Patient characteristics

We obtained data for 1,497 patients from which smoking status was available for 1,424 (95.1%) patients; 396 (27.8%) were smokers. Of all patients, 740 (49.4%) underwent endovascular treatment; 524 (35.0%) received mechanical thrombectomy alone and 216 (14.4%) patients received mechanical thrombectomy in combination with IA-thrombolysis. Median NIHSS on admission was 17 (Interquartile Range Limits [IQR] 14–21). These and other demographic and baseline clinical characteristics of all patients and according to smoking status are presented in **Table 1**.

**Table 1:** Baseline clinical characteristics of all patients, and according to smoking status.

	All patients	Smokers	Non-smokers
	(N = 1424)	(N = 396)	(N = 1028)
Age, Mean (±SD*)	65.5 (±13.7)	59.4 (±12.7)	67.8 (±13.4)
Sex, %female (n)	46.7% (699)	39.4% (156)	49.4% (508)
Cerebrovascular risk factors			
Atrial fibrillation, % (n)	23.7% (355)	16.2% (64)	28.1% (289)
Diabetes, % (n)	15.4% (230)	12.4% (49)	16.1% (165)
Hypertension, % (n)	55.0% (824)	45.7% (181)	58.2% (598)
Hyperlipidemia, % (n)	34.5% (517)	28.8% (114)	36.3% (373)
Myocardial infarction, % (n)	6.3% (95)	7.1% (28)	6.5% (67)
Coronary heart disease, % (n)	10.1% (151)	5.1% (20)	11.2% (115)
Congestive heart failure, % (n)	3.3% (49)	1.5% (06)	4.1% (42)
Prior stroke/TIA†, % (n)	10.6% (158)	7.1% (28)	12.1% (124)
NIHSS on admission, median (IQR‡)	17 (14–21)	17 (13–21)	17 (14–21)
Site of vessel occlusion			
Internal Carotid Artery (ICA) Only, % (n)	20.7% (202)	17.3% (43)	21.6% (143)
M1 segment only, ICA with involvement of M1 segment of Middle cerebral artery, % (n)	74.5% (729)	76.6% (190)	73.9% (489)
Single M2 segment only, % (n)	4.3% (42)	4.8% (12)	4.2% (28)
Other, % (n)	0.5% (05)	1.2% (03)	0.3% (02)
Endovascular Treatment, % (n)	49.4% (740)	50.3% (199)	48.9% (503)
Mechanical Thrombectomy only, % (n)	35.0% (524)	35.1% (139)	33.8% (347)
Mechanical thrombectomy + Intra-arterial thrombolysis, % (n)	14.4% (216)	15.2% (60)	15.2% (156)
Alteplase, % (n)	90.6% (1357)	93.4% (370)	89.2% (917)
Time to Endovascular treatment, median (IQR)	4.0 (3.05–4.91)	3.94 (3.16–4.76)	4.0 (3.0–4.93)

SD = standard deviation

†TIA = transient ischemic attack

‡IQR = interquartile range.

### Smokers versus non-smokers

Smokers were found to be, on average, younger in age (mean age, 59.4 ± 12.7 vs. 67.8 ± 13.4 years) and less commonly females (39.4% vs. 49.4%). Moreover, smokers were found to have less often a medical history of other cardiovascular risk factors like atrial fibrillation (16.2% vs. 28.1%), hypertension (45.7% vs. 58.2%), hyperlipidemia (28.8% vs. 36.3%), myocardial infarction (7.1% vs. 6.5%), coronary heart disease (5.1% vs. 11.2%), congestive heart failure (1.5% vs. 4.1%) or prior stroke/transient ischemic attack (TIA) (7.1% vs. 12.1%). Site of vessel occlusion or stroke severity on admission did not differ between groups. Distribution of mRS at 90 days was significantly lower in smokers compared to non-smokers (3 [IQR, 2–4] vs. 3 [IQR, 2–5]; p = 0.02). Smokers demonstrated higher BI (97.5 [IQR, 70–100] vs. 90 [IQR, 50–100]; p = 0.03), as well as lower mortality rates at 90 days (10% vs. 17.3%; p <0.001). Dichotomized endpoints based on mRS (good outcome and excellent outcome) did not differ between groups in univariate analysis (**Table 2**).

**Table 2:** Univariate analysis of primary outcome endpoints based on smoking status.

	Smoker	Non-smokers	p-value
*mRS day 90, median (‡IQR)	3.00 (2–4)	3.00 (2–5)	0.02
‡BI day 90, median (IQR)	97.5 (70–100)	90.0 (50–100)	0.03
Mortality at 3months, % (n)	10% (39)	17.3% (176)	0.00
Good outcome at 3 months, % (n)	42.3% (165)	38.8% (395)	0.23
Excellent outcome at 3 months, % (n)	23.3% (91)	23.9% (243)	0.83

* mRS = modified Rankin Score

†IQR = interquartile range

‡BI = Barthel Index.

### Generalized linear model for main outcome parameters

Smoking in itself had no clear effect on functional recovery (i.e. crude and adjusted RR of 0.97 [95% CI, 0.79–1.20] and 1.20 [95% CI, 0.89–1.62] for excellent outcome, **S1 Table**). Similar results were observed for the other primary endpoints when the analyses were restricted to those patients who underwent mechanical thrombectomy alone (i.e. adjusted RR of 1.0 [95% CI 0.84–1.28] and 1.1 [95%CI 0.78–1.46] for good and excellent outcome, respectively; **S1 Table**).

In the analyses amongst patients who underwent mechanical thrombectomy + IA-thrombolysis, point estimates of smokers—compared to non-smokers—were higher for excellent outcome three months post-stroke (adjusted RR of 1.65 [95% CI, 0.77–3.55]). Smokers had lower RR for mortality following mechanical thrombectomy + IA-thrombolysis in crude and adjusted analyses (crude RR 0.4 [95% CI 0.17–3.95] and adjusted RR 0.70 [95% CI, 0.33–1.48]; **Fig 1, S1 Table**).

**Fig 1:** Regression analysis of primary endpoints according to mode of therapy. Models were adjusted for the following covariates: age, sex, hypertension, atrial fibrillation, baseline NIHSS, and time to endovascular treatment.

### Interaction analysis of exposure variables (smoking + IA-thrombolysis)

Patients who underwent mechanical thrombectomy alone had significantly different cardiovascular risk profiles compared to patients who received mechanical thrombectomy + IA-thrombolysis; patients who had mechanical thrombectomy alone had less atrial fibrillation (21.7% vs. 28.7%), prior history of myocardial infarction (2.3% vs. 13.9%) and stroke (10.3% vs. 13.4%; **S2 Table**). Treatment with mechanical thrombectomy had an adjusted RR of 1.79 [95% CI, 1.46–2.21] for a good outcome. In comparison, treatment with mechanical thrombectomy + IA-thrombolysis (in reference to treatment with mechanical thrombectomy alone) was associated with a far less favorable outcome (i.e. adjusted RR of 0.56 [95% CI, 0.46–0.69]), most likely due to confounding by indication.

The crude mRS distributions in the four exposure categories shows patients in the two IA-thrombolysis categories had a less favorable mRS distribution compared to those who received mechanical thrombectomy alone. Median mRS of smokers + IA-thrombolysis was lower compared to non-smokers receiving IA-thrombolysis (median 3 [IQR 2–4] vs. median 4 [IQR 2–5.75]; p = 0.016) in univariate analysis.

In corresponding regression analyses presented in **Fig 2** (corresponding **S3 Table**), estimated RRs for all four categories in a combined exposure analysis are presented. Compared to those patients who neither received IA-thrombolysis nor smoke, smoking alone had no effect on outcome (**Figs 2 and 3**). Point estimates of smokers who received IA-thrombolysis were higher for favorable outcome (good and excellent outcome) than point estimates for non-smokers who received IA-thrombolysis. Smokers who received IA-thrombolysis had lower point estimates for mortality compared to non-smokers who received IA-thrombolysis (**S3 Table**).

**Fig 2:** Interaction analysis of smoking and mode of treatment. Interaction analysis based on presence of exposure variables (smoking and intra-arterial thrombolysis [IA-thrombolysis]), presenting crude and adjusted relative risk (RR). Reference category refers to non-smokers who received mechanical thrombectomy without IA-thrombolysis. The model is adjusted for the following covariates: age, sex, hypertension, atrial fibrillation, baseline NIHSS, and time to endovascular treatment.

**Fig 3:** Modified Rankin Scale distribution. Distribution of scores on the modified Rankin scale (mRS) in percentages among patients receiving endovascular therapy, according to exposure variables (smoking +/-) and intra-arterial thrombolysis added to mechanical thrombectomy (IAT +/-).

### Collateral status, recanalization, and reperfusion rates

In the subgroup analyses, collateral status, lesion progression (relative or absolute lesion growth), or recanalization status did not differ in univariate analysis between smokers and non-smokers. However, non-smokers had significantly higher reperfusion rates (11.6% vs. 6.8%) compared to smokers (**S4 Table**). We did not have sufficient data to study the effect of smoking who received IA-thrombolysis only treatment.

## Discussion

In this cohort of moderate to severe AIS patients enrolled in endovascular RCTs, smokers had significantly better outcomes in terms of functional recovery and mortality three months post-stroke compared to non-smokers in univariate analysis. Adjusted analyses indicated that the observed smoking paradox was largely explained by differences in baseline clinical risk profiles. In a focused analysis including only EVT patients, point estimates of smokers suggested better outcomes for smokers compared to non-smokers in patients receiving mechanical thrombectomy + IA-thrombolysis, however the estimates were not very precise.

Smokers were significantly younger, more often male, and had markedly fewer comorbidities (**Table 1**). In line with previous studies, smokers had a slightly better functional recovery three months post stroke in terms of mRS and BI as well as lower mortality rates compared to non-smokers in univariate analysis (**Table 2**) [2–4]. In a generalized linear model including all patients eligible for EVT regardless of intervention, smoking had no relevant effect on outcome parameters in adjusted analyses (i.e. adjusted RR of 1.1 [95% CI, 0.87–1.28]; p = 0.93 for good outcome; **Fig 1 and S1 Table**). The same was true in patients who underwent mechanical thrombectomy alone. Similar results were reported recently in the Taiwan Stroke Registry, which included approximately 89,000 subacute stroke cases [7]. This highlights the importance of the so-called index-event-bias [16, 17] of smokers due to their lower clinical risk profiles, particularly with respect to age.

In our combined exposure analysis (combination of smoking and IA-thrombolysis in four categories), IA-thrombolysis in non-smokers led to significantly reduced chances of a long-term favorable outcome (i.e. adjusted RR of 0.24 [95% CI, 0.14–0.41] for excellent outcome, and adjusted RR of 2.76 [95% CI, 1.74–4.37] for mortality) in comparison to non-smokers who received mechanical thrombectomy alone (reference category; **Fig 2 and S3 Table**). A possible explanation for this observation is that IA-thrombolysis is often used as a rescue therapy if mechanical thrombectomy cannot achieve full recanalization of the occluded vessel, and this is most likely the case in patients with severe cardiovascular comorbidities [18, 19]. However, the point estimates revealed that smokers fared better than non-smokers for all clinical outcome parameters in focused analysis of patients who received mechanical thrombectomy with IA-thrombolysis (**Figs 2 and 3**). A possible explanation for this beneficial effect of smoking may be increased recanalization rates in smokers following IA-thrombolysis resulting from increased efficacy of intra-arterial thrombolysis [3]. However, this effect could also be due to chance.

Authors have also hypothesized that the smoking paradox could be explained by increased collateralization due to chronic ischemia resulting from large artery atherosclerosis, which may hold ischemic tissue viable until reperfusion is achieved [20, 21]. Despite low numbers, we found no evidence for increased collateralization assessed on pre-treatment angiography in smokers in univariate analysis in this study (**S4 Table**).

In the current analyses non-smokers showed increased rates of reperfusion compared to smokers (11.6% vs. 6.8%; p<0.01), however data on recanalization and reperfusion was not available for our group of interest, namely smokers who received IA-thrombolysis. Further limitations of this study include missing data relevant to our research question i.e. type of smoking habits (i.e. type of tobacco consumption, pack years etc.) and IA-thrombolysis dosages to assess possible dose-effect on treatment efficacy, as well as stroke etiology to adjust for when assessing collateral status between smokers and non-smokers; other potentially relevant clinical parameters (such as body-mass-index, pre-stroke mRS, and site of arterial occlusion) also could not be adjusted for as these parameters were not commonly available. The latter is a limitation inherent to our study design, in which data was analyzed from pooled trial data not primarily designed to address our research question. We could not adjust for details of the study design in these analyses because trial data are provided in a blinded fashion to prevent re-analyses of completed RCTs. Lastly, some of our results could be chance findings. The consistency of the direction of the different observed effects suggests that this might not be the case. Still, given the broad confidence intervals, it is fair to say that strong conclusions regarding the effect estimates cannot be drawn and that the true effect of smoking on thrombolysis is actually clinically irrelevant. Nonetheless, this is the largest analysis of the smoking paradox yet in a homogenous cohort of patients with large vessel occlusions stemming from endovascular RTCs.

### Summary/Conclusions

In summary, in patients with proven vessel occlusion, tobacco smoking alone had no clear clinical effect on functional recovery post-stroke in our study. However in the analysis focused on patients who received IA-thrombolysis, consistent shifts in RRs of smokers indicate possible better functional outcomes and lower mortality rates in smokers, which is not entirely explicable due to index-event-bias of smokers alone (i.e. younger age and fewer comorbidities). Needless to say, smoking has well-known detrimental effects on the cardiovascular system and should be by no means encouraged.

## Supporting information

S1 Table Regression analysis of primary endpoints according to mode of therapy. (DOCX)

S2 Table Baseline clinical characteristics of patients with mechanical thrombectomy alone and in combination with IA-thrombolysis according to smoking status. (DOCX)

S3 Table Interaction analysis of smoking and mode of treatment. (DOCX)

S4 Table Univariate analysis of secondary outcome parameters based on smoking status. (DOCX)
